# Relationship between Changes in Blood Glucose and Blood Lipid Levels and the Risk of Thyroid Cancer in Patients with Type 2 Diabetes Mellitus

This article has been retracted.

**DOI:** 10.1155/2023/4814328

**Published:** 2023-04-11

**Authors:** Bowei Zhang, Zhe Song, Li Ren, Jinju Wang, Yi Gu, Chao Feng, Tong Liu

**Affiliations:** ^1^Department of Thyroid Surgery, Sichuan Provincial People's Hospital, University of Electronic Science and Technology of China, Chengdu, China; ^2^Chinese Academy of Sciences Sichuan Translational Medicine Research Hospital, Chengdu 610072, China

## Abstract

**Objective:**

To investigate the relationship between changes in blood glucose and blood lipid levels and the risk of thyroid cancer in patients with type 2 diabetes mellitus.

**Methods:**

A total of 159 patients with type 2 diabetes who were treated in our hospital between June 2018 and February 2021 were recruited and assigned into the observation group, including 136 patients with type 2 diabetes without thyroid cancer (nonthyroid cancer group) and 23 patients with type 2 diabetes complicated with thyroid cancer (thyroid cancer group), and 120 healthy subjects during the same period were selected as the control group. Glycated hemoglobin (HbAlc), total cholesterol (TC), triacylglycerol (TG), high density lipoprotein cholesterol (HDL-C), and low density lipoprotein cholesterol (LDL-C) were detected and compared. Pearson's method was conducted to analyze the correlation between serum HbAlc level and TC, TG, HDL-C, and LDL-C levels in patients with type 2 diabetes mellitus; multivariate logistic regression analysis was performed to analyze the influencing factors of thyroid cancer in patients with type 2 diabetes mellitus.

**Results:**

The serum HbAlc level and the incidence of thyroid cancer in patients with type 2 diabetes mellitus in the observation group were significantly higher than those in the control group (*P* < 0.05). The levels of TC, TG, and LDL-C in patients with type 2 diabetes mellitus in the observation group were significantly higher than those in the control group, and the level of HDL-C was significantly lower than that in the control group (*P* < 0.05). The correlation analysis showed that serum HbAlc levels in patients with type 2 diabetes were positively correlated with TC and TG levels and negatively correlated with HDL-C levels (*P* < 0.05) and not correlated with LDL-C levels (*P* > 0.05). Compared with the type 2 diabetes patients without thyroid cancer, the serum HbAlc, TC, and TG levels of the patients with type 2 diabetes mellitus in the thyroid cancer group were significantly higher, and the levels of HDL-C were significantly lower (*P* < 0.05). There was no significant change in the level of LDL-C (*P* > 0.05). Multivariate logistic regression analysis showed that serum HbAlc, TC, and TC levels were all risk factors for thyroid cancer in patients with type 2 diabetes mellitus (*P* < 0.05), while serum HDL-C level was a protective factor for thyroid cancer in patients with type 2 diabetes mellitus (*P* < 0.05).

**Conclusion:**

Thyroid cancer in type 2 diabetes patients may be linked to elevated levels of blood HbAlc, TC, and TG. HbAlc may raise the risk of thyroid cancer in type 2 diabetes patients by modulating blood lipid levels, which might serve as a marker to assess the risk of thyroid cancer in type 2 diabetes mellitus patients. However, since this study did not conduct in vitro and in vivo experiments, how HbAlc affects the pathogenesis of thyroid cancer has not been described in this study, which is also our future research direction. It is expected to provide new ideas for the prevention and treatment of thyroid cancer.

## 1. Introduction

Thyroid cancer (TC) and diabetes (DM) are both common diseases of the endocrine system. In the past 50 years, the global incidence of TC has continued to increase, and the disease is expected to become the fourth largest type of malignant tumor worldwide. TC is a malignant tumor originating from the follicular epithelial cells of the thyroid, and its histological classification includes papillary thyroid carcinoma (PTC), follicular thyroid carcinoma (FTC), medullary thyroid carcinoma, and anaplastic thyroid carcinoma, of which PTC is the most common subtype [1].

DM is a chronic metabolic disease characterized by elevated blood sugar. Epidemiological studies have found that the prevalence of TC in DM patients is significantly increased, and DM may increase the risk of TC. Current Western medicine treatment strategies include preventive screening and lifestyle interventions such as diet and exercise, drugs, and weight management. In addition to traditional oral drugs, Western medicine treatment includes dual-arc drugs, insulin secretagogues, and oral administration (for Gliban). These drugs demonstrate clear hypoglycemic effects yet are associated with side effects. Despite the intervention of Western medicine which can delay the progression of the disease and prolong their life to a certain extent, most patients might eventually die due to various complications.

According to the current epidemiological studies at home and abroad, compared with non-DM patients, the risk of TC in DM patients is significantly increased, indicating that DM and TC are correlated [2]. A prospective study based on a large sample of DM patients showed that the risk of TC in female DM patients was 1.46 times higher than that in non-DM women (95% CI: 1.01-2.10), and in women with differentiated TC, the risk of developing FTC was higher at PTC. A retrospective cohort study of 127 290 DM patients showed that the risk of TC was significantly increased in DM patients, and the risk was higher in males than in females (male: SIR = 1.83; 95% CI: 1.32-2.54; female: SIR = 1.40, 95% CI: 1.22-1.62). The prevalence of TC in patients with type 2 diabetes (T2DM) was also significantly higher than that in the non-T2DM group (OR = 1.89; 95% CI: 0.856-4.163), and the prevalence of TC in men with T2DM was significantly higher than that in women. Not only the prevalence of TC in patients with T2DM increases but also patients with TC and T2DM are more prone to cervical lymph node and distant metastasis than patients with TC alone. Therefore, it is of great significance to study the factors affecting thyroid cancer in patients with type 2 diabetes to control the progression of the disease and prevent its deterioration [3].

Glycated hemoglobin (HbAlc) is the product of the combination of blood glucose and hemoglobin, which can effectively reflect the recent glycemic control of patients with type 2 diabetes [4]. Dyslipidemia is intricately linked to the development of metabolic inflammation and insulin resistance, with elevated triglyceride-rich lipoproteins and lower high-density lipoprotein-cholesterol (HDL-C) being the major barriers that accompany insulin resistance in the liver. Excessive energy is generally stored under our skin, around our internal organs, and in our peritoneum in the form of fat. Blood lipids can be converted into fats and are the general term for lipid components in plasma, including triglycerides (TG), phospholipids, cholesterol, and free fatty acids (FFA). Lipids are fat-soluble and insoluble in water and must be combined with apolipoproteins in the blood to be transported in the blood and enter tissue cells. Lipoproteins are synthesized by the liver and are the form in which lipids are present, transported, and metabolized in the blood. In the event of that the exogenous uptake, endogenous synthesis, and lipoprotein synthesis, metabolism and transport of lipids in the body are hindered; it can lead to blood lipid metabolism disorders. Clinical studies have shown that the risk of thyroid cancer is closely related to the changes in blood sugar and blood lipid levels in patients. Long-term hyperglycemia and hyperlipidemia increases the incidence and risk of related cancers [5].

In addition to the development of bioinformatics, there has been a lot of accumulation of basic research data on diabetes, and there are also many predictive models for diabetes or thyroid cancer. Although these provide certain ideas, these are only predictions and have not been subjected to routine basic experiments or applied to patients. Therefore, clinical evidence-based evidence is also very important. Although many studies have shown that there is a relationship between diabetes and lipid metabolism, the clinical effect of HbAlc, total cholesterol (TC), low density lipoprotein cholesterol (LDL-C), high-density lipoprotein cholesterol (HDL-C), and triglyceride (TG) on thyroid cancer in patients with type 2 diabetes currently remains poorly understood [6]. Hence, the present study investigated the relationship between changes in blood glucose and lipid levels and the risk of thyroid cancer in patients with type 2 diabetes by detecting serum HbAlc levels and blood lipid levels of TC, TG, HDL-C, and LDL-C.

## 2. Materials and Methods

### 2.1. Participants

A total of 159 patients with type 2 diabetes who were treated in our hospital (Department of Thyroid Surgery) between June 2018 and February 2021 were recruited and assigned into the observation group, including 136 patients with type 2 diabetes without thyroid cancer (nonthyroid cancer group) and 23 patients with type 2 diabetes complicated with thyroid cancer (thyroid cancer group), and 120 healthy subjects during the same period were selected as the control group. There were 136 cases in this study (nonthyroid cancer group) and 23 cases of thyroid cancer. There exists a 6-fold gap, but our calculations based on references and sample size did not bias the results and conclusions of this study.

The original sample size calculation estimated that 100 patients in each group would be needed to detect a 3-point difference between groups in a 2-sided significance test with a power of 0.8 and an alpha error level of 0.05.

The trial was performed in accordance with standards of Good Clinical Practice and the Declaration of Helsinki. The trial protocol and all amendments were approved by the appropriate ethics (BI-HY20180203). All patients provided written informed consent before enrolment. The trial protocol has been published online and is available with the full text of this article.

The observation group included 79 males and 60 females; the mean age was 54.81 ± 9.48 years; the mean BMI was 23.68 ± 5.76 kg. There were 68 males and 52 females in the control group; the mean age was 54.73 ± 9.29 years; the mean BMI was 23.56 ± 5.81 kg. There was no significant difference in general data between the two groups of patients (Table 1).

### 2.2. Inclusion and Exclusion Criteria

Inclusion criteria are as follows: (1) patients who met the criteria of the American Diabetes Association; (2) thyroid cancer was confirmed by clinicopathological diagnosis; (3) the patients and their families were informed of the study and signed the informed consent; and (4) patients who can adhere to the treatment for at least 1 month and complete the main observation indicators.

Exclusion criteria are as follows: (1) patients with heart, lung, liver, and kidney insufficiency, infectious diseases, blood system diseases, autoimmune diseases, acute complications of diabetes, and severe mental disorders were excluded; (2) patients with primary thyroid cancer or other types of diabetes; (3) patients taking hormones and drugs that affect blood sugar and blood lipid levels; (4) patients with poor compliance and unable to cooperate with this study; and (5) complicated with severe infection, systemic immunological disease, uncontrolled unstable hypertension (resting blood pressure 5 140/90 mmHg and fluctuation over 20 mmHg within one week), severe cardiopulmonary insufficiency, severe acute and chronic diabetes complications, severe arrhythmia, surgery, trauma, peripheral vascular disease, abnormal organ function and serious primary diseases of the blood system, malignant tumors, and mental illness; (6) those with diabetic ketosis or severe infection in recent half month; and (7) pregnant or breastfeeding women.

### 2.3. Sample Collection and Index Detection

In the morning, 10 mL of fasting peripheral venous blood was drawn from the patient, placed in an EDTA tube and centrifuged at 3000 r/min at a low temperature of 4°C for 10 min, and the upper serum was drawn into a sterile EP tube; an automatic biochemical analyzer (purchased from Beckman Coulter Co., Ltd. Company, model: AU5800) was used to detect serum HbAlc, TC, TG, HDL-C, and LDL-C levels in patients.

### 2.4. Statistical Analysis

If the parameter beta is either a difference of means, a log odds ratio, or a log hazard ratio, then it is reasonable to assume that *b* is unbiased and normally distributed.

Statistical analysis was performed using the SPSS/Statistics 18.0 software for Windows (SPSS Inc., Chicago, IL). The paired *t*-test and chi-square test were performed to compare the differences in measurement data (*x*±*s*) and count data (*n* (rate)). Pearson method was used to analyze the correlation between serum HbAlc level and TC, TG, HDL-C, and LDL-C levels in patients with type 2 diabetes mellitus; multivariate logistic regression analysis was used to analyze the factors affecting patients with type 2 diabetes mellitus complicated with thyroid cancer. All statistical significance levels were set at a *P* value of less than .05.

## 3. Results

### 3.1. Serum HbAlc Levels and Incidence of Thyroid Cancer

The serum HbAlc level and the incidence of thyroid cancer in patients with type 2 diabetes mellitus in the observation group were significantly higher than those in the control group (*P* < 0.05, Table 2).

### 3.2. Blood Lipid Levels

The levels of TC, TG, and LDL-C in patients with type 2 diabetes mellitus in the observation group were considerably greater than those in the control group, whereas the level of HDL-C was significantly lower (*P* < 0.05, Table 3).

### 3.3. Correlation Analysis between Serum HbAlc Level and Blood Lipid Level in Patients with Type 2 Diabetes Mellitus

The correlation analysis showed that serum HbAlc levels in patients with type 2 diabetes were positively correlated with TC and TG levels and negatively correlated with HDL-C levels (*P* < 0.05) and not correlated with LDL-C levels (*P* > 0.05, Table 4).

### 3.4. Serum HbAlc Levels and Blood Lipid Levels in Patients with Type 2 Diabetes in Different Groups

Compared with the type 2 diabetes patients without thyroid cancer, the serum HbAlc, TC and TG levels of the patients with type 2 diabetes mellitus in the thyroid cancer group were significantly higher, and the levels of HDL-C were significantly lower (*P* < 0.05). There was no significant change in the level of LDL-C (*P* > 0.05, Table 5).

### 3.5. Multivariate Analysis of Thyroid Cancer in Patients with Type 2 Diabetes Mellitus

Taking the type 2 diabetes mellitus patients with thyroid cancer as the dependent variable and serum HbAlc, TC, TG, HDL-C, and LDL-C levels as independent variables, multivariate logistic regression analysis was performed. The results showed that serum HbAlc, TC, and TC levels were all risk factors for thyroid cancer in patients with type 2 diabetes mellitus (*P* < 0.05), while serum HDL-C level was a protective factor for thyroid cancer in patients with type 2 diabetes mellitus (*P* < 0.05, Table 6).

## 4. Discussion

China witnesses an incidence of diabetes of 10%, and it has become an epidemic disease from a rare disease, and the total figure in China has exceeded 100 million [7]. Type 2 diabetes constitutes the highest proportion of different types of diabetes, and it is associated with abnormal metabolism of blood glucose and blood lipids. Long-term abnormal metabolism of blood glucose and blood lipids can easily lead to lesions in different organ systems of patients, which further serves as a common risk factor for cancer lesions [8]. Thyroid cancer is a common clinical endocrine tumor, and its incidence has been on a rise in recent years, yet the clinical pathogenesis of thyroid cancer remains unclear [9]. Clinical studies have shown that the incidence of thyroid cancer in patients with type 2 diabetes can be 8 times higher than that in healthy individuals. These two diseases are both endocrine and metabolic disorders, so their pathogenesis may overlap. However, some clinical studies have shown that the level of tumor markers in patients with type 2 diabetes is not correlated with the presence of malignant tumors in the body [10]. Therefore, this study investigates the factors that affect the risk of thyroid cancer in patients with type 2 diabetes by observing the levels of blood glucose and blood lipids in patients with type 2 diabetes.

HbAlc is an important indicator for clinical monitoring of patients with type 2 diabetes. It is formed by the nonenzymatic sugar reaction between blood sugar and the amino acid terminal of serum hemoglobin. It has small biological variability and less detection requirements and is not easily affected by blood sugar fluctuations. It can effectively reflect the blood sugar status and blood sugar control of patients [11]. Scholar Noh et al. [12] have found that patients with long-term hyperglycemia usually have disordered thyroid secretion, which is more likely to form thyroid cancer than patients with normal blood sugar. A study by Qi et al. [13] pointed out that serum HbAlc levels in patients with type 2 diabetes are significantly correlated with thyroid hormone levels, and the imbalance of serum HbAlc levels in patients may lead to disorders of thyroid secretion. In the results of research by scholar Roh [14], it was found that the prevalence of thyroid cancer in the type 2 diabetes group was significantly higher than that in the control group, and the levels of blood glucose, serum HbAlc, blood lipids, and thyroid-stimulating hormone in type 2 diabetes patients complicated with thyroid cancer were higher than those in type 2 diabetes patients without thyroid cancer. It is believed that maintaining good blood sugar, serum HbAlc and blood lipid levels in patients with type 2 diabetes is helpful for the maintenance of thyroid function and the prevention of thyroid cancer [15].

Reportedly, serum HbAlc level is a risk factor for cancer in patients with type 2 diabetes [16]. It is also reported that blood glucose and blood lipid levels in patients with type 2 diabetes are closely related to the occurrence of thyroid cancer and thyroid autoimmune diseases [17], and the incidence of thyroid cancer and thyroid autoimmunity increases with the abnormal levels of blood sugar and blood lipids in patients [18]. Predictably, serum HbAlc and blood lipid levels in patients with type 2 diabetes may be related to the occurrence of thyroid cancer, but the specific mechanism is not yet clear [19].

In this study, we compared the levels of serum HbAlc, TC, TG, LDL-C, and HDL-C and the incidence of thyroid cancer in patients with type 2 diabetes mellitus and healthy subjects. The levels of TC, TG, and LDL-C and the incidence of thyroid cancer were higher than those of the healthy control group, while the HDL-C level was lower than that of the healthy control group. This shows that the changes of serum HbAlc and blood lipid levels are related to the occurrence of type 2 diabetes, and the risk of thyroid cancer in patients with type 2 diabetes is increased. However, whether the changes of serum HbAlc and blood lipid levels are involved in the development of thyroid cancer in patients with type 2 diabetes is elusive. Relevant studies have shown that serum thyroid-stimulating hormone (TSH) is positively correlated with PTC and PTC cervical lymph node metastasis. The clinical diagnosis of PTC and lymph node metastasis and the research on the diagnosis and treatment of the disease have different degrees of biological and medical research value [20, 21]. Additionally, TSH also participates in the regulation of blood lipid levels, and the concentration of non-HDL-C and TG may increase with the increase of its concentration, and the concentration of HDL-C may decrease. It indicates that TSH may be involved in the regulation of blood lipid metabolism, acting independently of TH, and contrary to the effect of TH, that is, TSH can fight hyperlipidemia at lower levels, while TSH at higher levels will increase the risk of hyperlipidemia [22]. Clinically, it is found that in majority of patients, one or more abnormal liver function and blood lipid indexes are observed in the examination of liver function and blood lipids.

The serum HbAlc level in patients with type 2 diabetes is positively correlated with the levels of TC and TG but negatively correlated with the level of HDL-C; this indicates that there is an interaction between the level of serum HbAlc and blood lipid levels, which may jointly be involved in the complications of patients with type 2 diabetes mellitus [23]. Afterwards, we compared the levels of serum HbAlc, TC, TG, LDL-C, and HDL-C in patients with type 2 diabetes mellitus without thyroid cancer and those with thyroid cancer. The level of TG was significantly higher than that of patients without thyroid cancer, while the level of HDL-C was significantly lower than that of patients without thyroid cancer. It is speculated that the changes of serum HbAlc and blood lipid levels may be the influencing factors of thyroid cancer in patients with type 2 diabetes mellitus. Serum HbAlc, TC, and TG levels were all influencing factors for thyroid cancer in patients with type 2 diabetes mellitus, while serum HDL-C level was a protective factor for thyroid cancer in patients with type 2 diabetes mellitus. This shows that serum HbAlc and blood lipid levels are related to thyroid cancer in patients with type 2 diabetes mellitus, and increased serum HbAlc, TC, and TG levels and decreased serum HDL-C levels are associated with an increased risk of thyroid cancer [24, 25]. Regarding the clinical efficacy, Hb, MCHC, MCV, and adverse reactions and other indicators, this study did not find significant differences. Therefore, no special analysis was performed. It may be attributed to the fact that this study is a single-center experiment, and only patients in this region were included, and the patient's constitution and living habits may have a certain impact. In addition, only 159 patients with diabetes were included in this study, of which only 23 patients had thyroid cancer, and there was a certain weight offset in this proportion.

Inevitably, this study also has certain limitations. First, this trial is a retrospective study, and there is a lack of analysis of other exposure information, such as smoking history, drinking history, iodine environment, physical activity level, waist-to-hip ratio, blood pressure, and other factors. The influence of these confounding factors on the results cannot be excluded. Second, many relevant literatures at home and abroad have shown that insulin resistance is closely related to the pathogenesis of thyroid cancer. Additionally, insulin resistance, as the central link of metabolic syndrome, may be the common mechanism of abnormal glucose and lipid metabolism and blood lipids involved in the pathogenesis of thyroid cancer. The relationship between insulin resistance and thyroid cancer is very important. Since this study is a retrospective study, the data are collected from patients undergoing thyroid surgery. Before surgery, only blood glucose, blood lipids, and thyroid function were routinely detected, but insulin levels were not detected, and the correlation between insulin resistance and thyroid cancer could not be explored. In the future, a prospective study on the relationship between insulin resistance and thyroid cancer will be carried out. Third, the data of this study were taken from June 2018 and February 2021, mainly based on the ultrasound results, surgery on thyroid nodules of category 4a and above (TI-RADS classification), which may lead to a higher rate of surgery for benign nodules, but in 2020. After January 2018, the hospital has stipulated that patients with thyroid nodules of category 4a and above (TI-RADS classification) detected by ultrasound routinely undergo preoperative FNA examination, and the operation rate of benign nodules has been significantly reduced. In addition, the glucose and lipid metabolism indexes and BMI levels collected in this study are only preoperative levels and cannot reflect the duration of each index in patients before surgery. Therefore, subsequent studies at the cellular and molecular level need to be conducted to further explore the relationship between glucose and lipid metabolism indicators, uric acid and BMI, and the occurrence and development of thyroid cancer, so as to provide new ideas for clinical prevention and treatment of thyroid cancer. Although there are some shortcomings, this method provides certain ideas for judging thyroid cancer and can be applied to routine observation and prediction of thyroid patients in various medical institutions.

To sum up, thyroid cancer in patients with type 2 diabetes may be related to the increased levels of serum HbAlc, TC, and TG. HbAlc may increase the risk of thyroid cancer in patients with type 2 diabetes by regulating blood lipid levels, which could serve as a marker to evaluate the risk of thyroid cancer in patients with type 2 diabetes mellitus. Although no specific mechanism was investigated in this study, no specific biological genetic targets were tested. However, this study provides a certain evidence-based basis for future basic experiments and drug design and provides a certain direction for new epigenetic targets for clinical treatment and diagnosis of thyroid cancer. In the future, the studies with larger sample size will be conducted, and in vitro and in vivo experiments will be carried out to confirm the mechanism.

## Figures and Tables

**Table 1:** Comparison of general data of the two groups of patients (*n* (%)).

	Observation group (*n* = 159)	Control group (*n* = 120)	*t*/*x*^2^	*P*
Gender			0.001	0.978
Male	79	68		
Female	60	52		
Mean age (year)	54.81 ± 9.48	54.73 ± 9.29	0.07	0.944
Mean BMI (kg/m^2^)	23.68 ± 5.76	23.56 ± 5.81	0.172	0.864

**Table 2:** Comparison of serum HbAlc levels and incidence of thyroid cancer between the two groups of patients (*x* ± *s*).

Groups	*n*	HbAlc	Thyroid cancer incidence (%)
Observation group	159	9.33 ± 2.95	23 (14.5%)
Control group	120	5.72 ± 1.87	2 (1.7%)
*t*/*x*^2^	—	11.74	13.732
*P*	—	<0.001	<0.001

**Table 3:** Comparison of blood lipid levels in the two groups of patients (*x* ± *s*, mmol/L).

Groups	*n*	TC	TG	HDL-C	LDL-C
Observation group	159	5.53 ± 1.07	2.72 ± 0.89	1.15 ± 0.31	3.22 ± 0.95
Control group	120	4.25 ± 0.88	1.80 ± 0.53	1.62 ± 0.47	2.86 ± 0.77
*t*	—	10.661	10.055	-10.045	3.394
*P*	—	<0.001	<0.001	<0.001	0.001

**Table 4:** Correlation analysis between serum HbAlc level and blood lipid level in patients with type 2 diabetes mellitus.

Variables	TC	TG	HDL-C	LDL-C
HbAlc				
*r*	0.442	0.476	-0.488	0.366
*P*	0.016	0.001	0.001	0.142

**Table 5:** Comparison of serum HbAlc levels and blood lipid levels in patients with type 2 diabetes in different groups (*x* ± *s*, mmol/L).

Groups	*n*	HbAlc	TC	TG	HDL-C	LDL-C
Non thyroid cancer group	136	9.07 ± 2.79	5.47 ± 0.76	2.65 ± 0.73	1.20 ± 0.36	3.20 ± 0.88
Thyroid cancer group	23	10.47 ± 3.11	5.95 ± 1.12	3.08 ± 0.94	0.75 ± 0.21	3.44 ± 1.02
*t*	—	-2.189	-2.596	-2.5	5.82	-1.182
*P*	—	0.03	0.01	0.013	<0.001	0.239

**Table 6:** Multivariate analysis of influencing factors of thyroid cancer in patients with type 2 diabetes mellitus.

Variables	*B*	SE	Wald	*P*	OR	95% CI
HbAlc	0.804	0.488	2.711	0.001	2.233	1.525-3.271
TC	0.360	0.235	2.347	0.026	1.433	1.228-1.673
TG	0.808	0.512	2.492	0.002	2.244	2.203-2.286
HDL-C	-0.561	0.358	2.452	0.015	0.571	0.441-0.739
LDL-C	0.140	0.119	1.393	0.258	1.151	0.869-1.524

## Data Availability

All data generated or analyzed during this study are included in this published article.
